# Balance Analysis of Peripheral Neuropathy in Type 2 Diabetes Mellitus Based on Logistic Regression Equation

**DOI:** 10.1155/2022/2113758

**Published:** 2022-05-18

**Authors:** Lixin Zhang, Qianqian Du, Manman Yao, Mai Wang, Bing Ge

**Affiliations:** ^1^Nursing Department, The Second Hospital of Shijiazhuang, Hebei 050000, China; ^2^Department of Endocrinology, The Second Hospital of Shijiazhuang, Hebei 050000, China; ^3^Department of Obstetrics and Gynecology, The Second Hospital of Shijiazhuang, Hebei 050000, China; ^4^Pediatrics Department, The Second Hospital of Shijiazhuang, Hebei 050000, China

## Abstract

This paper analyzes the factors of peripheral neuropathy in type 2 diabetes mellitus and puts forward a balanced analysis of peripheral neuropathy in type 2 diabetes mellitus based on logistic regression equation. A total of 1192 eligible patients were selected as the study subjects. All selected patients underwent 75 g oral glucose tolerance test to measure fasting blood glucose and insulin and 2-hour postprandial blood glucose and 2-hour postprandial insulin, as well as neuroelectrophysiological examination. The results showed that the OR values of age, course of disease, fingertip blood glucose immediately after admission, and 2-hour blood glucose were greater than 1, and the *P* values were all less than 0.05, which were the risk factors of diabetic peripheral neuropathy. OR value of *β* cell function index (HBCI) is less than 1. *P* is less than 0.05, and it is a protective factor of diabetic peripheral neuropathy. Laboratory indicators are as follows: 75 g OGTT: 0-hour blood glucose, 2-hour blood glucose, and glycosylated hemoglobin; serum creatinine; glutamate transaminase; fibrinogen; ten items of hemoglobin; and indexes reflecting islet function: islet *β* is thin, and there are significant differences in cell function index, insulin resistance index, and insulin secretion index between the non-DPN group and DPN group. Age, course of disease, fingertip blood glucose immediately after admission, and blood glucose within 2 hours after admission were the risk factors for diabetic peripheral neuropathy. Islet *β* cell function index (HBCI) is a protective factor of diabetic peripheral neuropathy.

## 1. Introduction

Diabetic neuropathy refers to the damage of the nervous system caused by chronic hyperglycemia of diabetes and various pathophysiological changes caused by it, which can affect any part of the whole nervous system. It is one of the common and serious complications of diabetes and can affect 50%-90% of diabetic patients [1]. The most common diabetic neuropathy is peripheral neuropathy, the pathogenesis of this disease is complex, and its clinical manifestations are varied. It can not only occur in the late stage of diabetes, but also, 8% of newly diagnosed diabetic patients have found neuropathy [2]. Diabetic peripheral neuropathy is a hidden, gradual, and slow process, which is nonspecific and difficult to reverse. It is an important risk factor for diabetic foot and other critical diseases. It is the most common cause of nontraumatic amputation. Once diabetic patients have neuropathy, it is extremely difficult to treat them [3]. If we can find diabetic peripheral neuropathy early, actively and effectively control blood sugar and give symptomatic treatment [4], and carry out some necessary foot care, serious consequences such as ulcer, gangrene, and amputation of the foot may be avoided [5]. In view of this research problem, Younger and others reported that the course of diabetes is the influencing factor of DPN [6]. Studies by Dixit et al. show that hyperglycemia is one of the most important causes of DPN. Effective control of hyperglycemia in the early stage of DPN can regenerate the nerve fibers that have lost their functions and restore some functional fovea. However, if hyperglycemia is not well controlled for a long time, it will lead to irreversible damage of the peripheral nerve, which will gradually worsen [7]. Malone found that abnormal insulin signal may be an important initiating factor of DPN and play an important role in the occurrence and development of DPN [8]. On the basis of the current research, this paper proposed the balance analysis of peripheral neuropathy in type 2 diabetes based on logistic regression equation. The results showed the analysis of influencing factors of peripheral neuropathy in elderly patients with type 2 diabetes, the baseline age and disease course; fingertip blood glucose immediately upon admission; laboratory indicators: 75 g OGTT: 0 h blood glucose, 2 h blood glucose, and HbA1c; serum creatinine; alanine aminotransferase; and fibrinogen. There were significant differences in 10 items of hemoglobin and the indexes reflecting the function of shadow islet: islet *β*-cell function index, insulin resistance index, and insulin secretion index in non-DPN group and DPN group (*P* < 0.05). Further multifactor analysis showed that the influencing factors of senile type 2 diabetic peripheral neuropathy included age, course of disease, blood glucose 2 hours after meals, fingertip blood glucose immediately after admission, and islet *β* cell function index.

## 2. Methods

### 2.1. Research Object

All the inpatients in the Department of Endocrinology and Geriatrics of the Staff General Hospital of a coal-fired power group company selected 1216 eligible elderly patients with type 2 diabetes, of which 24 were rejected because of incomplete data, and 1192 patients with complete data were selected as the research objects. All selected patients were tested by 75 g oral glucose tolerance test for fasting blood glucose, insulin, blood glucose, and insulin at 2 hours after meal and nerve electrophysiological examination. The youngest is 60 years old, and the oldest is 87 years old, with an average of 65.82±5.98 years old. There were 768 males (64.43%) and 424 females (35.57%) [9].

Inclusion criteria were as follows: confirmed type 2 diabetes (according to WHO 1999 diagnostic criteria) and age ≥ 60 years old.

Exclusion criteria were as follows: type 1 diabetes mellitus; patients with secondary diabetes; oral or inhaled corticosteroids were used during hospitalization or for a long time; and users of antipsychotic drugs.

### 2.2. Laboratory Inspection Items

Glycosylated hemoglobin (HbA1c); immediate fingertip blood glucose at admission; 75 g oral glucose tolerance test (OGTT): FPG, 2hPG, FINS, and 2hINS; total cholesterol (TC), triglyceride (TG), high-density lipoprotein-cholesterol (HDL-C), low-density lipoprotein-cholesterol (LDC-C); glutamate transaminase (ALT); total bilirubin (TBIL), conjugated bilirubin (DBIL); blood urea nitrogen (BUN) and serum creatinine (Cr); fibrinogen (FIB); and white blood cells (WBC), red blood cells (RBC), and platelets (PLT) were 19 items [10].

### 2.3. Neuroelectrophysiological Examination

The results of neuroelectrophysiological examination were collected, and the examination instrument was NDI-500P+ (Poseidon) neuroelectrodiagnostic instrument. The method of nerve electrophysiological examination was 18-9: specific measurement: motor nerve conduction velocity (MCV) and motor nerve action potential (CMAP) amplitude of the left and right median nerve (elbow→wrist), ulnar nerve (elbow→wrist), tibial nerve (popliteal→medial malleolus), and common peroneal nerve (below knee); sensory nerve conduction velocity (SCV) and sensory nerve action potential (SNAP) amplitude of median nerve (middle finger→wrist), ulnar nerve (little finger→wrist), peroneal nerve (lateral malleolus→calf); F wave; and H reflex.

### 2.4. Diagnosis and Exclusion Criteria of Diabetic Peripheral Neuropathy

For the diagnostic criteria of diabetic peripheral neuropathy (DPN), neuroelectric physiological examination is the “gold standard” to diagnose DPN, specifically

1. a clear history of diabetes
2. neuropathy occurring during or after diagnosis of diabetes
3. the clinical symptoms and signs are consistent with the manifestations of diabetic peripheral neuropathy
4. two or more items of nerve conduction velocity (NCV) slowed down

The diabetic peripheral neuropathy (DPN) exclusion criteria are as follows:

1. Neuropathy caused by other causes, such as spinal neuropathy, nutritional deficiency, liver and kidney diseases, paraneoplastic syndrome, connective tissue diseases, and genetic diseases
2. History of taking drugs (isoniazid, furazolidone) that can cause peripheral nerve damage and exposure to some toxic substances (such as heavy metals), anticholinergic drugs, and drugs that may affect autonomic main nerve function
3. Diseases that can cause subjective sensory disorders (such as hysterical sensory disorders) and unable to cooperate with the inspection, such as low intelligence and difficult to understand
4. Patients with special type diabetes and type 1 diabetes

### 2.5. Grouping

According to the results of neuroelectrophysiological examination (NET), 1192 hospitalized elderly patients with type 2 diabetes were divided into a simple diabetes group (non-DPN) and diabetic peripheral neuropathy group (DPN).

### 2.6. Statistical Analysis

All the data were verified and entered into the computer and analyzed by SPSS 16.0 statistical software. The measurement data were described by the standard deviation of mean soil,$\bar{x}\pm s$, using variance analysis. Chi-square test was used for counting data (*x*^2^ test). Logistic regression analysis was used for multivariate analysis (*P* < 0.05 was statistically significant) [11].

### 2.7. Logistic Regression Equation

In logistic regression model analysis, some methods of variable screening can be used to control multicollinearity, and the logarithm of each value can be used to establish a general linear regression model of *INX* over *InX*_1_, *InX*_2_ ⋯ *InX*_6_.

## 3. Results and Analysis

### 3.1. Analysis of Influencing Factors of DPN in Elderly Patients with Type 2 Diabetes Mellitus

1. The influence of age, course of disease, body mass index, and blood pressure on DPN

The analysis of variance showed that the average age, course of disease, and body mass index of patients in the non-DPN group were 63.33 ± 4.46 years, 2.69 ± 3.12 years, and 24.93 ± 4.12 kg/m^2^, respectively. The mean systolic blood pressure was 125.60 ± 30.41 mmHg, and the mean diastolic blood pressure was 79.21 ± 51.18 mmHg. In the DPN group, the average age was 66.64 ± 6.18 years, the average course of disease was 8.10 ± 6.42 years, and the average body mass index was 24.55 ± 4.4.35 kg/m^2^. The mean systolic blood pressure was 127.59 ± 38.73 mmHg, and the mean diastolic blood pressure was 75.0 ± 42.48 mmHg. Compared with the non-DPN group, the DPN group was older (*F* = 71.83, *P* = 0.001) and had a longer course of disease (*F* = 193.67, *P* = 0.001), and the difference was statistically significant. There was no significant difference in BMI, SBP, and DBP (*P* > 0.05) [12].

(2) The influence of gender and smoking on DPN

The chi-square test showed that there were 196 males (66.7%) and 98 females (33.3%) in the non-DPN group. In the DPN group, there were 572 males (63.7%) and 326 females (36.3%). There were 184 smokers in the non-DPN group, accounting for 62.59% of non-DPN patients, and 579 smokers in the DPN group, accounting for 64.48% of DPN patients. Different genders (*x*^2^ = 0.85, *P* = 0.356) and smoking or not (*x*^2^ = 0.34, *P* = 0.556) were not statistically significant between the non-DPN group and DPN group (*P* > 0.05) [13].

(3) The influence of blood sugar on DPN

The analysis of variance showed that the fingertip blood glucose (11.1 ± 4.72 mmol/L), fasting blood glucose (9.11 ± 2.52 mmol/L), 2-hour blood glucose (15.79 ± 6.46 mmol/L/L) and glycosylated hemoglobin (9.62 ± 2.55%) in the DPN group immediately after admission. Compared with the two groups, the indexes of blood glucose control in the DPN group were significantly worse than those in the non-DPN group, including fingertip blood glucose (*F* = 53.80, *P* = 0.001), fasting blood glucose (*F* = 121.19, *P* = 0.001), 2-hour blood glucose (*F* = 64.12, *P* = 0.001), and glycosylated hemoglobin (HbA1c). The difference was statistically significant [14].

(4) Effects of blood lipid and uric acid on DPN

The analysis of variance showed that the total cholesterol, triglyceride, high-density lipoprotein-cholesterol, and low-density lipoprotein-cholesterol in the DPN group were5.64 ± 16.19 mmoL/L/L, 2.11 ± 3.63 mmol/L, 1.21 ± 0.66 mmol/L, and 3.28 ± 7.71 mmol/L, respectively. Compared with the two groups, there was no significant difference in the total cholesterol (*F* = 0.008,*P* = 0.927), triglyceride (*F* = 0.011,*P* = 0.916), high-density lipoprotein-cholesterol (*F* = *l*.100,*P* = 0.294), and low-density lipoprotein-cholesterol (*F* = 0.965).

(5) Influence of liver function and kidney function on DPN

Analysis of variance showed that in the non-DPN group, the concentration of alanine aminotransferase was 25.84 ± 20.98 IU/L and the concentration of total bilirubin was 17.23 ± 7.92 *μ*mol/L, the concentration of conjugated bilirubin was 3.53 ± 2.72 *μ*mo1/L, and blood urea nitrogen concentration was 6.28 ± 4.23 mmol/L. Islet Β Cell function index and insulin resistance index represent the effects on diabetes nephropathy. Analysis of variance showed that islets in the DPN group Β Cell function index was 42.68 ± 41.62, insulin resistance index was 4.11 ± 4.63, insulin secretion index was 1.12 ± 1.05, insulin sensitivity index was 0.02 ± 0.02, islet Β Cell function index *F* = 54.633 (*P* = 0.001), and insulin secretion index *F* = 15.327 (*P* = 0.001), and the above indexes were lower than those in the DPN group. In the DPN group, alanine aminotransferase (29.13 ± 18.73 IU/L/L), total bilirubin (17.03 ± 7.34 *μ*mol/L/L), combined bilirubin (3.93 2.93 *μ*mol/L), blood urea nitrogen (6.37 2.72 mmol/L), serum creatinine (78.07), and serum creatinine (*F* = 7.248, *P* = 0.007) reflecting renal function were higher than those in the non-DPN group, and the difference was statistically significant (*P* < 0.05). There was no significant difference in total bilirubin (*F* = 0.343, *P* = 0.558), conjugated bilirubin (*F* = 0.282, *P* = 0.596), and urea nitrogen (*F* = 1.977, *P* = 0.16) [15].

(6) The effects of leukocyte, hemoglobin, platelets, and fibrinogen on DPN

Analysis of variance showed that the DPN group had leukocytes (6.63 ± 2.84) × 10^9^/L, hemoglobin 154.10 ± 44.84 g/L, platelet (190.41 ± 67.85) × 10^9^/L, and fibrinogen 4.02 ± 1.92 g/L. Compared with the two groups, the DPN group had higher WBC (*F* = 0.328, *P* = 0.567), but there was no significant difference between the two groups. The fibrinogen was high (*F* = 8.458, *P* = 0.004), and the difference between the two groups was statistically significant. Hemoglobin was low (*F* = 6.422, *P* = 0.011), and the difference between the two groups was statistically significant. Platelet was low (*F* = 1.356, *P* = 0.245), and there was no statistically significant difference between the two groups (*P* > 0.05).

(7) The effects of islet *β* cell function index and insulin resistance index on DPN. ANOVA showed that the islet *β* cell function index (42.68 ± 41.62), insulin resistance index (4.11 ± 4.63), insulin secretion index (1.12 ± 1.05), and insulin sensitivity index (0.02 ± 0.02) in the DPN group and the islet *β* cell function index (*F* = 54.633,*P* = 0.001) and insulin secretion index (*F* = 15.327,*P* = 0.001) were lower in the DPN group, and the differences between the two groups were statistically significant. The DPN group had higher insulin resistance index (*F* = 11.276, *P* = 0.001), and the difference was statistically significant. Insulin sensitivity index (*F* = 0.919, *P* = 0.338) showed no significant difference between the two groups

### 3.2. Stratified the Age, Course of Disease, and Glycosylated Hemoglobin Affecting Diabetic Peripheral Neuropathy and Understood Its Influence on DPN

1. The influence of different ages on DPN

The chi-square test showed that the incidence of DPN was 6.5% in the 60-year-old group, 30.4% in the 60-64-year-old group, and 53.1% in ≥65 groups (*x*^2^ = 65.621, *P* = 0.001); with the increase of age, the incidence of DPN increased gradually, and there were statistical differences between the two groups in three age groups (*P* < 0.05) (see Figure 1 for details).

(2) The influence of different courses of disease on DPN

The chi-square test showed that the incidence of DPN was 27.6% in the group with a course of less than 3 years, 34.7% in the group with a course of 3-9 years, and 37.6% in the group with a course of more than 10 years (*x*^2^ = 2.301*E*2, *P* = 0.001), suggesting that with the prolongation of the course of disease, the incidence of DPN increased significantly, and there was a statistical difference between the two groups (*P* < 0.05), as shown in Figure 2 [16].

(3) Effects of different glycosylated hemoglobin on DPN

The chi-square test showed that glycosylated hemoglobin was divided into three layers, and the incidence of DPN increased with the increase of glycosylated hemoglobin (*x*^2^ = 37.01, *P* = 0.001), and there was a statistical difference between the two groups (*P* < 0.05) (see Figure 3 for details).

### 3.3. Multivariate Logistic Regression Analysis of DPN in Type 2 Diabetes Mellitus

In the analysis of logistic regression model, sometimes, the multicollinearity can be controlled by variable screening. In addition to deleting the independent variable f that has no significant impact on the dependent variable *Y*, several variables that have a significant impact on the dependent variable *Y* can also be screened from the collinear relationship of group A variables to overcome the problem of collinearity. In order to use the forward method, the OR values of age, course of disease, fingertip blood glucose immediately after admission, and blood glucose within 2 hours should be greater than 1. However, for some practical problems, even if there is collinearity between independent variables, it is still expected to establish the regression between *Y* and a given independent variable. The general linear regression model of *INX* to *InX*_1_, *InX*_2_ ⋯ *InX*_6_ is established by the logarithm of each value, as shown in the following formula:

(1) $$\begin{array}{c} InY=InA+\alpha {InX}_{1}+\beta {InX}_{2}+\gamma {InX}_{3}+\theta {InX}_{4}+\lambda {InX}_{5}+\omega {InX}_{6}. \end{array}$$

In order to further analyze the influence of the above factors on diabetic peripheral neuropathy, the presence or absence of diabetic peripheral neuropathy (none = 0, yes = 1) was taken as dependent variable, and the age, course of disease, immediate fingertip blood glucose, fasting blood glucose, 2-hour blood glucose and glycosylated hemoglobin at admission, serum creatinine, glutamate transaminase, fibrinogen, hemoglobin, the 13 influencing factors of islet cell function index, insulin resistance index, and insulin secretion were analyzed by multivariate logistic regression. According to the standard of*a* = 0.05, forward method was selected for analysis. As a results, the OR values of age, course of disease, fingertip blood glucose immediately after admission, and blood glucose within 2 hours are greater than 1, and the *P* values are all less than 0.05, which are the risk factors of diabetic peripheral neuropathy. The OR value of *β* cell function index (HBCI) is less than 1; *P* is less than 0.05, which is the protective factor of diabetic peripheral neuropathy [17] (as shown in Table 1).

### 3.4. Peripheral Neuropathy in Elderly Patients with Type 2 Diabetes Mellitus Is the Result of Comprehensive Influence of Many Factors

DPN is the result of many factors. The main risk factors include age, sex, waist-hip ratio, course of disease, blood glucose drift, postprandial blood glucose, and low income. However, there are relatively few large sample studies on the elderly. In this study, when analyzing the influencing factors of peripheral neuropathy in elderly patients with type 2 diabetes mellitus, we found that the patient's age, course of disease, immediate fingertip blood glucose at admission, 2-hour blood glucose, glycosylated hemoglobin, serum creatinine, glutamic transaminase, fibrinogen, hemoglobin, and the indicators reflect islet function. This study found that elderly patients with type 2 diabetes peripheral neuropathy were affected by the following factors: first, compared with those in hospital, OGTT fasting blood glucose in patients with diabetes was relatively stable; for blood glucose after intervention, the result may be low and the impact on DPN may be reduced. Islet *β* is thin, and there are significant differences in cell function index, insulin resistance index, and insulin secretion index between the non-DPN group and DPN group (*P* < 0.05). And further multifactor analysis, the influencing factors of peripheral neuropathy in elderly patients with type 2 diabetes include age, course of disease, blood glucose 2 hours after meal, fingertip blood glucose immediately after admission, and islet *β* cell function index [18].

### 3.5. Age and the Incidence of DPN

The results of this study showed that the incidence of DPN was 75.34%. With the increase of age, the incidence of DPN increased gradually, which was 6.5% in 60-year-old group, 30.4% in 60-64-year-old group, and 53.1% in ≥65 groups. The abnormal rates of motor nerve conduction velocity (MNCV) and sensory nerve conduction velocity (SNCV) in patients with type 2 diabetes were 71.76% and 58.47%, respectively. 28% of 70-79 years old and 35% of ≥80 years old suffered from peripheral neuropathy. Aging can decrease the function of islet *β* cells in rats. Age is an independent risk factor for DPN. With the increase of age and the prolongation of disease course, the function of islet *β* cells gradually declines, which leads to the related complications of diabetes. Middle-aged and elderly people have become a high-risk group of diabetes due to the increase of age and genetic and environmental factors. However, during the development of glucose metabolism disorder, the function of islet *β* cells decreased gradually.

### 3.6. Incidence of Fingertip Blood Glucose and DPN Immediately after Admission

The results showed that fingertip blood glucose, fasting blood glucose, 2-hour blood glucose, and glycosylated hemoglobin were all risk factors of peripheral neuropathy in elderly patients with type 2 diabetes mellitus. Step-by-step multivariate logistic regression analysis showed that fingertip blood glucose was the risk factor of peripheral neuropathy in elderly patients with type 2 diabetes immediately after admission. The reasons were analyzed: immediate fingertip blood glucose can better reflect the out-of-hospital blood glucose control status of patients and represents the normal blood glucose control level. However, the long-term blood glucose control status is involved in the occurrence and development of peripheral neuropathy in type 2 diabetes mellitus. In related studies, there are few studies on immediate fingertip blood glucose and diabetic complications, but as a means of monitoring blood glucose, because its convenience, simplicity, popularity, and operability are of great help to clinical practice. Dynamic blood glucose detection (CGMS) has good correlation, accuracy, and consistency with venous blood glucose and fingertip blood glucose.

### 3.7. Incidence of Blood Glucose and DPN 2 Hours after Meal

The results showed that OGTT 2-hour blood glucose was significantly correlated with DPN, which was a risk factor for diabetic peripheral neuropathy. Compared with young patients, elderly patients may have abnormal action of dual hormones with organ degeneration, that is, decreased insulin secretion and delayed peak insulin secretion after meals, while glucagon does not decrease, resulting in continuous increase of postprandial blood sugar. After 2 hours, it still increased significantly or reached its peak. According to the comprehensive analysis of the influence of blood sugar on DPN, whether it is fingertip blood sugar immediately after admission or blood sugar 2 hours after meals, the mechanism of DPN is still oxidative stress caused by hyperglycemia.

### 3.8. Influence of Other Factors on the Incidence of DPN

In this study, not in multivariable logistic regression analysis, it was found that in fasting plasma glucose and the elderly with type 2 diabetes peripheral neuropathy, the following factors were considered: first, the fasting blood sugar for diabetes patient is relatively stable after OGTT fasting glucose, in contrast to the hospital at that time; for the blood sugar of blood glucose after intervention, the result may be on the low side, and the effect on DPN is reduced. In addition, compared with fasting state, postprandial state lasts longer, so postprandial blood glucose may be more involved in the occurrence and development of DPN. In this study, no relationship was found between smoking and peripheral neuropathy in the elderly with type 2 diabetes. The reasons for this analysis were as follows: smoking was not stratified during data statistics, and only smoking was considered. Therefore, the influence of smoking on complications was ignored.

## 4. Conclusion

In this paper, a balanced analysis of peripheral neuropathy in type 2 diabetes mellitus based on logistic regression equation was proposed, and 1192 patients with complete data were selected as research objects. After testing and analyzing the related items, the results show that in the analysis of influencing factors of peripheral neuropathy in elderly patients with type 2 diabetes, the baseline age and course of disease; immediate fingertip blood glucose at admission; laboratory indicators: 75 g OGTT: 0-hour blood glucose, 2-hour blood glucose, and glycosylated hemoglobin; serum creatinine; glutamate transaminase; fibrinogen; ten items of hemoglobin; and indexes reflecting islet function: islet *β* is thin, there are significant differences in cell function index, insulin resistance index, and insulin secretion index between non-DPN group and DPN group (*P* < 0.05). Further multifactor analysis showed that the influencing factors of senile type 2 diabetic peripheral neuropathy included age, course of disease, blood glucose 2 hours after meals, fingertip blood glucose immediately after admission, and islet *β* cell function index.

## Figures and Tables

**Figure 1:** Relationship between age and DPN.

**Figure 2:** Relationship between course of disease and DPN.

**Figure 3:** Relationship between HbA1c and DPN.

**Table 1:** Multivariate logistic regression analysis of diabetic peripheral neuropathy.

Influence factor	*B*	SE	Wald	*P* values	The OR value
Course of disease	0.257	0.024	103.933	0.001	1.233-1.35
Fingertip blood glucose immediately upon admission	0.11	0.026	17.112	0.001	1.061-0.178
2-hour postmeal blood glucose	0.098	0.024	15.264	0.001	1.052-1.161
HBCI	-0.006	0.002	13.833	0.001	0.991-0.998

## Data Availability

The data used to support the findings of this study are available from the corresponding author upon request.
